# Potential of grid-connected decentralized rooftop PV systems in Sweden

**DOI:** 10.1016/j.heliyon.2023.e16871

**Published:** 2023-06-01

**Authors:** Tianqi Ruan, Monika Topel, Wujun Wang, Bjorn Laumert

**Affiliations:** Department of Energy Technology, KTH Royal Institute of Technology, Brinellvägen 68, Stockholm, 11428, Sweden

**Keywords:** Decentralized PV system, Grid networks, Techno-economic analysis, Swedish contexts, Urban areas

## Abstract

Solar power generation in Sweden is far from required capacity to help with transition towards 100% renewables in the power sector by 2040. Decentralized PV system attracts attentions given the conflicts of future increasing demands and land scarcity in the urban areas. However, it is not easy to implement it due to challenges on local conditions and lack of references.

This paper aims to propose an overview of the potential of small-scale grid-connected PV systems in a Swedish context and offer an example for urban PV system planning in Sweden or high latitude areas. A model considering weather, space, infrastructures and economics is developed and implemented with a real case in the Swedish context.

The findings verify the technical and economic feasibility of urban decentralized rooftop PV systems in the Swedish context. It is found that this kind of system does have considerable power potential in the Swedish context without land requirements. This kind of PV system could be a promising option for future power generation which satisfies part of demands and reduces pressure on external grids. The full potential could be only achieved with improved infrastructures, and the profitability of the system relies heavily on market and political conditions. This study can be a refence for other high latitude areas.

## Highlights

• The study considers weather, space, infrastructure conditions and economics.
• Distributed rooftop PV has big power potential but is limited by infrastructure.
• The system is economically feasible in Sweden but sensitive to market and policies.
• It provides a reference on urban PV integration for other high latitude areas.

## Abbreviations

PV: Photovoltaic
IEA: International Energy Agency
LCA: Life Cycle Analysis
GHG: Greenhouse Gas
KPIs: Key Parameter Indicators
SMHI: Swedish Meteorological and Hydrological Institute
LoD: Level of Detail
VAT: Value Added Taxes
SEK: Swedish Krona
CAPEX: Capital expenditure
OPEX: Operating expenditure
NPV: Net Present Value
SD: Standard Deviation

**Symbols**
$f_{i_{elle_{com}}}$: Ellevio charge fees for electricity consumption [öre/kWh]
$f_{i_{\_elle\_pro}}$: Ellevio charges for production [öre/kWh]
$f_{i_{bix}}$: Bixia charge fees for production/consumption [öre/kWh]
${CAPEX}_{unit}$: Capital expenditure per unit [SEK/kWp]
${OPEX}_{i}$: Operating expenditure of the i-th year [SEK]
${O\&M}_{fixed}$: Annual fixed operational and maintenance fees per unit [SEK/kWp/year]
$r_{s}$: Rate of subsidy [%]
$r_{e}$: Escalation rate [%]
$r_{d}$: Interest rate [%]
$I_{\max}$: Maximum current through the lines [A]
P: Power [W]
U: Voltage [V]
fp: power factor [−]
TB: Total benefits [SEK]
CaR: CAPEX reduction [SEK]
$B_{i}$: Benefits of the i-th year [SEK]
${CoR}_{i}$: Cost reduction due to self-consumption of the i-th year [SEK]
${Earn}_{i}$: Earnings from electricity export of the i-th year [SEK]
$C_{i\_elle}$: Cost reduction from Ellevio of the i-th year [SEK]
$C_{i\_bix}$: Cost reduction from Bixia of the i-th year [SEK]
sur: Surcharges for electricity consumption with Bixia [öre/kWh]
$E_{i\_com}$: Electricity consumption reduction of the i-th year [kWh]
$B_{i\_elle}$: Benefits from Ellevio of the i-th year [SEK]
$B_{i\_bix}$: Benefits from Bixia of the i-th year [SEK]
$E_{i\_pro}$: Electricity exported of the i-th year [kWh]
${Range}_{\min}$: The minimum value of the range [kW]
${Range}_{\max}$: The maximum value of the range [kW]
${Production}_{avg}$: Average power of PV production in a certain hour [kW]
${SD}_{pro}$: Standard deviation of PV production [kW]
${Loads}_{avg}$: Average power of loads in a certain hour [kW]
${SD}_{load}$: Standard deviation of loads [kW]

## 1 Introduction

### 1.1 Background

It is well established that conventional fossil-fuel based generation needs to be phased out due to its negative impacts on the environment and its non-renewability. Within this context, supported by policy and target requirements, the transition to renewable energy technologies has become an important focus to several countries across the world [1,2]. Many countries have set goals to reach carbon neutrality by 2045 or 2050 [3]. To achieve this, renewable energy technologies will contribute more on energy security in the future.

In recent years, photovoltaic (PV) power generation technologies are being integrated in the electricity system and constitute an increasing share of the power capacity. As the costs of PV panels decrease, decentralized rooftop PV systems have developed rapidly and are predicted to grow further in the future due to global transition to sustainability [4]. According to a survey by the International Energy Agency (IEA), many countries participate in research projects regarding grid-connected PV, including Spain, Germany and Sweden [5]. And some countries have already provided economic support for the decentralized PV systems, for example, the US and Australia give feed-in tariffs to consumers and it is found dramatic grow in PV installations [6].

In 2017, Sweden introduced ambitious climate policies and is currently a frontrunner country in the transition towards sustainability. The country set the goal to have net zero greenhouse gas emissions by 2045 [7] and to have a 100% renewable electricity production by 2040 [8]. Even though there are no specific targets for the development of PV, it is still expected that PV systems in Sweden will flourish in the long run from this political conditions [9]. By the end of 2019, PV installations reached more than 700 MW, of which almost 50% are residential ones [9]. Since the prices of 10.13039/501100013891PV systems continue to decrease along with political support of tax reduction or subsidy for initial costs, PV markets attract more public interests especially private individuals and small companies. However, the integration of solar power in the Swedish electricity system amounts today to only 0.4%, which is far away from the prediction by International Energy Agency and the Swedish Energy Agency that 5%–10% of electricity demands will be satisfied by PV production in 2040 [9,10].

It is not straightforward to implement decentralized PV systems in Sweden. Among the identified challenges for PV integration in Sweden there is the inherent dependence on local conditions since the performance of the PV systems fluctuate due to its dependence on weather. There would be a significant fluctuation of solar radiation, and thus PV production, in the different seasons. Moreover, there is an evident seasonal mismatch between PV production and electricity demand. In summer, when the loads are at their lowest level, the PV production surpasses the demand, while in winter, when loads are its highest, the PV systems produce little to no electricity. It is more expensive to keep stable output within these conditions. Another challenge is related to the limitation on existing infrastructure and scarcity of space in urban areas, both of which constrain the PV capacity due to limited installation. Due to scarcity of space for installation, the PV system is restricted and uncertain to meet the demands. In addition, integration of new PV system may put pressure on current grid network leading to overloading problems when the self-consumption in low (during summer). However, private individuals with increasing environmental awareness are still curious about the real potential of this grid-connected residential rooftop PV system in Sweden. The opportunities are already there, but it remains unknown if the full potential of PV systems could be achieved by overcoming the barriers. It is therefore very important to investigate and identify the barriers of decentralized PV integration in Sweden.

This study estimates the feasible power potential of PV system in a Swedish context. The study will focus on the urban decentralized grid-connected PV systems on the reference-case of Hammarby Sjöstad, a neighborhood located in southern Stockholm. Through the local citizen-driven initiative “*ElectriCITY”*, the district of Hammarby currently has higher environmental goals than the city of Stockholm and initiatives related to the introduction of smart energy systems are on-going. With the goal *Climate-neutral Sjöstaden 2030*, the district actively participates in innovative research and projects. Therefore, Hammarby is interesting and suitable for this study [11]. The study considers weather conditions, space restrictions and existing infrastructure limitations. The capacity of PV systems is calculated in Swedish weather conditions. The size of PV system is determined by space or gird network to investigate feasibility of full potential. The study intends to help decision makers to better plan for the target of 100% renewable energy production by 2040 and further net zero by 2045 and provides insights for residents to encourage participation in sustainable actions.

### 1.2 State-of-the-art

There are many studies regarding integration of PV technologies with urban grid networks. Zhang et al. [12] evaluated rooftop PV potential of different types of roof in Wuhan, China with conclusion that industrial, commercial, public and education units has highest potential and reaches more than 2000 GW h per year. The study specifically focused on power potential assessment without considering the impacts on demands and grid. Kanters and Horvat [13] quantified urban solar potential of buildings in Lund, Sweden especially concentrating on geometry impacts. The study confirmed the contribution of urban solar power to increasing renewable energy proportion but also focused mainly on power potential calculation rather than consider the whole electricity network. Yang et al. [14] evaluated rooftop solar potential at municipal and national level in a Swedish context and illustrated significant potential of solar power in Sweden. Similarly, the paper provided detailed research in generation and capacity while does not mention feasibility. Corcelli et al. [15] offered comprehensive life-cycle analysis (LCA) for rooftop PV system presenting environmental benefits with considerable reduction on greenhouse gas (GHG) emissions while regardless of technical and economic performance. Haegermark et al. [16] looked into economic aspect with Swedish cases implying the importance of political supports also presenting the impacts electricity demands and fuse size have on PV system performance. Since economic performance is of priority, the system is optimized based on profitability instead of technical limitations. The techno-economic perspective of building-mounted PV energy system in a Swedish context was analyzed in Ref. [17] where a comprehensive research on its processes and application, as well as evaluation of integration with heating systems is provided. However, the work performed in Ref. [17] did not comprise electricity grid network considerations. A case study analysis on urban energy systems, also based on Hammarby, was performed in Ref. [18]. Although the analyses mainly focused on district heating and heat pumps rather than PV systems, the research provided insights on modelling approaches and processes.

Spatial analytics started to assist system planning and design at many different fields in recent years, including energy system design. ArcGIS as a tool with comprehensive spatial analyzing methods occurs in many research regarding urban PV systems. Bayrakci Boz et al. [19] with the help of ArcGIS and light detection and ranging found the potential and feasibility of roof top solar power in Philadelphia, USA. Alhamwi et al. [20] modelled a GIS-based platform to find out feasibility and effectiveness of urban power systems with storage. Fonseca et al. [21] performed an optimization model referring cases in Switzerland to improve urban energy distribution and increase renewable sources integration with residential buildings. Choi et al. [22] utilized PV analyst in ArcGIS with TRNSYS to simulate and assess PV arrays and irradiation components.

Power flow analysis is commonly used for PV system planning. There are several studies regarding power flow analysis of grid-connected PV systems. Wang et al. developed a model of large–scale PV system to explore methods of power flow analysis [23]. The study involved PV system as case study while the main purpose is methodology of power flow analysis, rather than applications. Similarly, Juarz et al. also worked on algorithm part, and they deep into component level investigating on the control and operation of different processes [24]. Power flow analysis is also used for integration capacity improvement. Alsafasfeh et al. developed a model for optimal integration of large-scale PV system considering voltage fluctuation [4]. In addition, Lindberg et al. studied on site selection of large-scale PV park in Sweden involving combination of GIS technologies and power flow analysis [25]. The study put emphasis on spatial limitations.

In short, urban rooftop PV systems have been attracting worldwide attention recently. The PV systems are highly dependent on location, methods and results from other regions may fail to represent the performance of Swedish case. Even though there are research cases in Sweden, the analysis was performed from different perspectives: some considered large-scale system; and some looked into only one dimension among technical, environmental or economic aspects. Multi-perspective evaluation gives a more comprehensive overview of the system, the combination of different dimensions should be engaged, which was aimed in this present study.

With increasing force from land use and population, micro-grid starts to be a focus and requires more information on how the grid network operates with renewable sources on small scale. Studies that integrate spatial tools and power flow analysis tools arose increasingly within PV research in recent years. This paper evaluates system level with combination of ArcGIS and pandapower. The former one assists on spatial availability whereas the latter one copes with power flow analysis and grid limitations.

### 1.3 Aim and objectives

This paper provides an overview of the potential of small-scale grid-connected PV systems in a Swedish context and explores the impacts of barriers. The potential is assessed considering space, grid limitations, loads and economics. This paper aims to offer an example for urban PV system planning in Sweden. The analysis considers the combination of multiple dimensions with a more comprehensive evaluation. The study validates the feasibility of urban distributed solar system in high-latitude areas, and the method can be extended to other cases.

## 2 Methodology

In this section, the processes and methods involved in the study will be described in detail. The study begins with data collection regarding weather, buildings, PV panels and existing grid network. The data is gathered from respective relevant databases. The data is then used in the models created, including one for grid networks (grid model), one for PV production estimation (PV power model) and one for matching buildings and grid (spatial model). They are interconnected with each other. The whole designed system is structured by combination of these models. It is then simulated through power flow analysis and the results are assessed from technical and economic aspects. The whole processes are presented in Fig. 1, where data collected are in black rectangles, models and methods in green rectangles, outputs from models in black dash rectangles and key performance indicators (KPIs) in the green ellipse. More details are presented in the following sections.

**Fig. 1:** Processes of the study.

### 2.1 Data collection

#### 2.1.1 Weather data

In the study, the weather data of 2020 in Stockholm is gathered from Swedish Meteorological and Hydrological Institute (SMHI). The data is helpful to measure the available irradiations. To show the variation, hourly data is chosen. In this study, besides direct irradiation, diffuse irradiation and reflection irradiation are also considered.

#### 2.1.2 Building data

The building data is collected from open database of Stockholm City. The level of detail (LoD) of the building is at LoD 200, and due to this limitation, the rooftops are assumed to be flat. In total, there are 277 buildings included in this study.

#### 2.1.3 PV panels

The type of PV panels chosen is commonly and commercially available in Swedish PV market. It is assumed to be 300 Wp, and the size is 1 m × 1.7 m. All PV panels will be installed in the same fixed tilt angle. The distance between each line of the PV panels is assumed to be 2.4 m [4]. The efficiency is assumed to be 17%, as average commercial PV panels have this efficiency [4]. Beside basic conversion efficiency, the performance of PV panels is also influenced by the environment. In this study, the influence from environment such as temperature and dust are considered. Altogether it is assumed to be 10% loss including such as soiling, wiring and availability [26]. Reduction for obstacles and shading effects is 10% and 15% respectively [27]. The PVs will be installed on the rooftop of the buildings and operate for 20 years.

#### 2.1.4 Electricity grid

The grid network information is gathered from the grid operator. The data contains 2 grid networks including information of substations, distribution lines and measured loads. All these facilities already exist in the district, so the information is similar to real operation. In Hammarby, there are in total 19 substations and 2 external grid to support daily demands.

#### 2.1.5 Electricity contracts

The electricity fees in Sweden contain mainly two part-the costs to electricity network operators and to electricity trading companies. In this study all consumers in the district are connected to Ellevio AB as grid operator and the study assumes all contracts with Bixia for electricity trading, since it is widely accepted in Stockholm and provides renewable energy options.

According to the contracts for variable prices of Ellevio and Bixia, Table 1 lists the prices including taxes (VAT) measured by Swedish official currency-krona (SEK) and öre. According to the variable price contract with Ellevio, both electricity transfer fee and production incentives have two prices-high price time and other time. High price time refers to the period from 6 a.m. to 10 p.m. between November 1st and March 31st [28]. As for Bixia, except for fixed fee paid by month once signing the contract, charge, surcharge and electrical certificate are all related to electricity consumption. The charge fee changes according to the spot price of Nord Pool. The extra electricity is also sold based on the hourly spot price of Nord Pool. In this study, monthly spot price is used instead. And Table 2 lists the monthly average spot price in 2020 and 2021.

**Table 1:** Details on electricity tariffs and prices.

Contract	Description		Costs	Unit
Electricity network (Ellevio) [28,29]	Electricity transfer including VAT ($f_{i_{\_elle\_com}}$)	Normal time	11.00	[öre/kWh]
		High price time	62.5	
	Production including VAT ($f_{i_{\_elle\_pro}}$)	Normal time	2.70	
		High price time	3.50	
Electricity trading (Bixia) [30]	Consumption	Charge ($f_{i\_bix}$)	(Table 2)	
		Surcharge	4.00	
		VAT	25	[%]
	Production	Charge	(Table 2)

**Table 2:** Nord Pool monthly spot price in 2020 and 2021 [31].

Month	Price 2020	Price 2021	Unit
January	250	491	[SEK/MWh]
February	195	536	
March	150	368	
April	98	337	
May	135	435	
June	249	403	
July	93	591	
August	347	671	
September	348	918	
October	230	648	
November	241	835	
December	316	670	

#### 2.1.6 Costs for the PV system

In order to measure the economic performance of the system, information on Swedish PV system costs is collected. The initial costs for the whole system establishment (CAPEX), including components and installation, are dependent on the size of the system. Operation and maintenance costs of the i-th year (${OPEX}_{i}$) is estimated to be annual fixed cost (${O\&M}_{fixed}$) with an escalation rate ($r_{e}$) per year. With the system operating and becomes older, it is harder to keep the capacity and requires more for fixing. The interest rate in Sweden is set as 3% [17]. The tax for self-consumption decides on the size of the PV modules. Thanks to the new regulations from Swedish Energy Agency, the systems smaller than 500 kw are exempted from tax payment. In order to encourage transition to renewable energy sources, Swedish government offers subsidy on the modules and installation reducing 15% costs for materials and installation [32]. Table 3 summarizes the cost factors of PV system in Sweden.

**Table 3:** Parameters of PV module costs.

Parameter		Value	Unit
${CAPEX}_{unit}$ [9]	0–10 kW_p_	14.29	[SEK/W_p_]
	10–50 kW_p_	11.7	
	50–200 kW_p_	10.12	
	>200 kW_p_	7.5	
Capital reduction subsidy ($r_{s}$) [33]		15	[%]
${O\&M}_{fixed}$ [34]		50	[SEK/kW_p_/year]
Escalation rate of $\left(r_{e}\right)$ [34]		1	[%]
Interest rate ($r_{d}$) [17]		3	[%]

### 2.2 Models

#### 2.2.1 PV power model

The fixed tilt angle decides the amount of irradiation possibly received by PV panels. In order to measure the potential of the system, the PV panels will be installed with an optimal angle that received maximum annual irradiation. The optimal angle is calculated by varying the tilt angle from 0 to 90° and selecting the one that yields the maximum total irradiation on PV panels. Along with PV information, the power potential of each PV panel can be calculated. It is one of main parameters for assessing potential PV production. There are some assumptions for calculating the total available irradiation:

• All PV panels are assumed to orient towards due south since Stockholm locates in the northern hemisphere.
• All PV panels are considered to have unified position with same solar elevation as differences of longitude and latitude are negligible.
• The direct normal irradiance is set as zero when the incident angle between sun's ray and the normal of the PV panels is larger than 90°. In this case, the sunlight illuminates on the back of PV panels.
• Diffuse radiation is all regarded as isotropic due to the uncertainty of circumsolar calculation methods during the period of sunrise and sunset [7].
• The surrounding conditions are quite complicated and uncertain within the district. The ground is assumed to be horizontal and of infinite extent. It reflects solar beam isotopically.
• The reflectivity of the ground is set as the common value, 0.2.

In this study, hourly weather data for the whole 2020 is used to find the optimal tilt angle, and the peak reaches 37.0° with corresponding maximum annual feasible irradiation at 1.086 MW h/m^2^. The value is used for PV power calculation. The area value of each rooftop is obtained and adapted from the building data, which determines the size of PV system on each rooftop. Along with information of PV panels and calculated irradiation values, PV production of each building can be estimated.

#### 2.2.2 Spatial model

The collected building and electricity grid data contains geo-information. According to the location of buildings and grid line distribution, the buildings are sorted and matched with corresponding substations with assistance of ArcGIS. Thus, the PV systems on the rooftop are distributed into different substations. Each substation then has an influencing area, shown as Fig. 2. The PV production of each substation can be calculated as the sum of production from every building within the influencing area.

**Fig. 2:** Overview of the district and the influence area of each substation.

#### 2.2.3 Power flow analysis

The electricity grid in Hammarby Sjöstad can be subdivided into two parts, both of them containing several lines and substations. Each substation links with several lines that connect with buildings. Measured load data is aggregated at the level of substations. The grid is structured as shown in Fig. 3. Each substation links with some buildings and the PV systems are installed on the rooftops.

**Fig. 3:** Detailed structure of the PV model in the whole district.

The system is then built and simulated in power flow analysis tool, pandapower. Two different scenarios are analyzed and compared. The first is aiming at maximum utilization of all rooftop areas (scenario 1) and the other one takes limitations of existing infrastructure into account (scenario 2). There is no limitation on infrastructures set for scenario 1 which represents an improved infrastructure conditions where the loading is acceptable for the grid network. On the other hand, scenario 2 considers the impacts of line-overloading problem representing the current situation. It occurs when the real power flow exceeds the limitation for the lines [35]. In this study, the thresholds for line-overloading are set as 100%. For the lines, the maximum current flow is limited by the apparent power P, voltage U and power factor fp (equation (1)). In a Swedish context, power factor is set as 0.972 [36].

(1) $$I_{\max}=\frac{P}{U*fp*\;\sqrt{3}}$$

### 2.3 Techno-economic analysis

#### 2.3.1 Technical performance

Several indicators are chosen to check the technical performance for both scenario 1 and 2: solar fraction, self-consumption, self-sufficiency and export potential. Solar fraction refers to the ratio of total PV production to the total amount of loads; self-consumption represents the proportion of PV production that consumed; and self-sufficiency means the percentage of loads fulfilled with PV production [37]. During the period that PV production is higher than the loads, the residue part of electricity is capable for export to sell. The proportion of this part of electricity in total production is expressed as export ratio in this study. The inter-relationship of these 4 indicators will be evaluated for both scenario 1 and 2. They will also be compared between two scenarios to investigate the impacts of different conditions.

#### 2.3.2 Economic performance

In this study, the economic performance of the PV system will be mainly measured in two indicators-total benefits (TB) and net present value (NPV). These two parameters are relevant with CAPEX and OPEX. CAPEX is paid only in the first year (equation (2)), while OPEX accumulates year by year. The total OPEX is obtained by equation (3).

TB consists of two parts: initial capital reduction (CaR) and the sum of annual benefits during the whole lifetime (equation (4)). The annual benefits in the i-th year ($B_{i}$) includes cost reduction due to less electricity consumption (${CoR}_{i}$) and gains from electricity export (${Earn}_{i}$). CaR comes from the Swedish government who intends to support renewable energy systems. It depends on the total CAPEX and capital reduction subsidy ($r_{s}$) provided, as equation (5). According to section 2.1.5, ${CoR}_{i}$ should include cost reduction from Ellevio ($C_{i\_elle}$) and that from Bixia ($C_{i\_bix}$), as equation (6). Since the fixed fees are always paid, these two parameters are relevant with respective variable charges. The charge of Ellevio for production and consumption at different periods is fixed; however, the charge for Bixia changes according to electricity market. And a surcharge (sur) is required for consumption. With a certain amount of electricity consumption reduction ($E_{i\_com}$), the fees are calculated with equations (7), (8) for Ellevio and Bixia part respectively. Similarly, the gains from these two companies ($B_{i\_elle}$ and $B_{i\_bix}$ respectively) are calculated based on exported electricity ($E_{i\_pro}$), as equations (9), (10), (11).

NPV is the sum of costs and benefits over the whole lifetime (equation (12)). It implies whether the investments would be paid back. Profitability is positively associated with the NPV value. If the value is greater than zero, it means the costs will be paid back in the end.

(2) $$CAPEX=Size*\;{CAPEX}_{unit}$$

(3) $$OPEX=\sum_{i=1}{OPEX}_{i}=\sum_{i=1}\frac{{O\&M}_{fixed}\;*{\left(1+r_{e}\right)}^{i-1}}{{\left(1+r_{d}\right)}^{i}}$$

(4) $$TB=CaR+\sum_{i=1}B_{i}=CaR+\sum_{i=1}\frac{{CoR}_{i}+{Earn}_{i}}{{\left(1+r_{d}\right)}^{i}}$$

(5) $$CaR=CAPEX*\;r_{s}$$

(6) $${CoR}_{i}=C_{i\_elle}+C_{i\_bix}$$

(7) $$C_{i\_elle}=E_{i\_com}*f_{i_{\_elle\_com}}\;*\left(1+VAT\right)$$

(8) $$C_{i\_bix}=E_{i\_com}*\left(f_{i\_bix}+sur\right)*\left(1+VAT\right)$$

(9) $${Earn}_{i}=B_{i\_elle}+B_{i\_bix}$$

(10) $${B_{i\_elle}=E}_{i\_pro}*f_{i_{\_elle\_pro}}*\left(1+VAT\right)$$

(11) $$B_{i\_bix}=E_{i\_pro}*f_{i\_bix}*\left(1+VAT\right)$$

(12) $$NPV=\sum_{i=0}\left(CAPEX+OPEX+TB\right)$$

## 3 Results and discussion

### 3.1 Technical performance

#### 3.1.1 Scenario 1

Based on the inputs listed in section 2.1 and 2.2, scenario 1 assumes all available space on the rooftops is fully utilized. The area available for solar production of each building has already been modified according to the solar map from Stockholm city. According to the division and assumption above for PV installation limitation, the potential area for PV installation and annual production at each substation are summarized in Fig. 4. Most substations have around 3000–7000 m^2^. Substation 3 has the smallest area, which is less than 1000 m^2^ while substation 7 has the largest area which is almost reaching 8000 m^2^. The annual solar production within the district has been estimated. It is more than 12 000 MW h. The trend line presents that PV production is positively relative to potential area and has the same trends. This is because only spatial limitation is considered in scenario 1.

**Fig. 4:** PV production in each substation influencing area for scenario 1.

Integration of the PV system changes the electricity distribution in the district. Fig. 5 presents the relationship of self-consumption and self-sufficiency with solar fraction (orange dots and blue dots respectively). Each dot represents a substation, some dots are labeled in the figure. The x-axis is solar fraction. Except substation 9a where solar fraction is larger than 100%, all other substations have the value smaller than 30%. For most of the substations, new PV systems could not provide enough electricity to meet the demands and there is a huge gap requiring external grid.

**Fig. 5:** Relationship between indicators of each substation for scenario 1– self-consumption (orange dots) and self-sufficiency (blue dots). (For interpretation of the references to color in this figure legend, the reader is referred to the Web version of this article.)

Self-consumption is mostly close to 100% at low solar fraction varying between 90% and 100%. With lower solar fraction, solar generation is so small that is always less than loads, so almost all electricity generated is used. Sometimes, loads become very low, for example during the summer vacation. Therefore, there might be some period when generation is higher than loads, so that self-consumption is not 100%. When solar fraction becomes larger, it is more likely to generate surplus electricity during the noon, and self-consumption ratio decreases. But as solar fraction is lower than 30%, self-consumption ratio remains higher than 90%. One exception is substation 9a. PV generation is higher than loads during operation periods, therefore, the self-consumption is much lower than the others, at around 30%.

In general, self-sufficiency increases with increasing solar fraction. With a certain load, higher solar fraction represents higher solar generation, and more part of loads can be met by the solar modules. However, self-sufficiency stays at a low percentage. Even solar fraction at around 120%, self-sufficiency is only 35%. PV system can only generate electricity during the day while more demands happen in the evening. As there is no storage equipment in the system, most demands are supported by an external grid. For the district, installing PV modules could help reduce dependence on external grid and increase the proportion of renewable energy to some extent, but not total independence and 100% renewable sources in the current context.

Fig. 6 shows the relationship of export ratio and self-consumption. Generally, higher self-consumption implies a lower export ratio, since more electricity is used within the influencing areas. 18 out of 19 substations can sell the extra electricity, except substation 13 with 100% self-consumption and 0 export ratio. The potential among different substations differs a lot. For example, substation 9a potentially exports more than 250 MW h electricity which takes up approximately 70% of total production; while other substations use majority of the electricity that PV modules produce for own loads less than 15% of total production can be sold. Half of them export between 50 and 100 MW h and the rest are lower than 20. This is because sometimes at noon when solar irradiation is quite high, there are several hours that the production is larger than the loads at that moment, especially in the summer. During the weekends or vacation when loads become stable and low, energy produced is potential to not only meet the needs but also to export. However, this period only occupies a smart part of the whole year thus the amount of surplus electricity is limited. If this part of electricity is utilized, further reduction on the grid consumption is more likely to achieve as well as energy independence, no matter for late use during night hour or export to other substations.

**Fig. 6:** Exported energy and self-consumption of each substation for scenario 1.

Fig. 7 shows seasonal average production and load variations of all substations within the day. Fig. 7a to d represent 4 seasons from spring to winter, respectively. The values for different substations vary a lot, so standard deviation (SD) of both production and loads are calculated (shown as shade in the figures). The load is always higher than the production in spring, autumn and winter, even with highest production and lowest loads, which confirms the low solar fraction. However, in the summer, when production is at peak, the production line transgresses the average loads line. It represents that the system gains extra electricity for export after meeting the demands in this condition. Comparing different seasons, the curves have similar trends within in the day for both production and loads. But the PV system operation period is different. In the summer, the systems are able to operate more than 15 h but half in the winter. Considering the value, production and loads are opposite. Loads are higher in the winter and lower in the summer, while production is larger in the summer and relatively small in the winter. Overall, there is a huge gap between production and loads, which requires external grid. It is also noted that the curves of production and loads do not match: the peak of loads arise later than production, which makes the system more difficult to operate as desired.

**Fig. 7:** Variations of power and loads within typical days of different seasons: (a) spring; (b) summer; (c) autumn; (d) winter.

Fig. 8 displays an example in summer and winter that the huge difference among different substations. Substation 9a (largest export ratio) and 13 (the only one without export potential) are chosen. Fig. 8a presents the curves of both PV power generation and loads of substation 9a in summer (left) and winter (right), and Fig. 8b presents those of substation 13. Substations with very low loads have large export potential even though the production is not the highest. In some substations, PV system operates at considerable power, but there is a huge gap between loads and production. The power is similar at approximately 220 kW, but the export potential is significantly different due to huge variation on loads. This is the reason for Fig. 7 is deceiving.

**Fig. 8:** Examples of different daily variation in summer and winter: (a) substation 9a; (b) substation 13.

Thus, Table 4 summarizes the difference between average production and load value (production minus load, maximum value) of each substation in summer and winter. The possible range is also calculated as following:

(13) $${Range}_{\min}=\min\left[\left({Production}_{avg}-{SD}_{pro}\right)-\left({Loads}_{avg}+{SD}_{load}\right)\right]$$

(14) $${Range}_{\max}=\max\left[\left({Production}_{avg}+{SD}_{pro}\right)-\left({Loads}_{avg}-{SD}_{load}\right)\right]$$

In summer, there are 4 stations with positive average value, but only four negative values for maximum values. It implies that in summer most substations are possibly potential to export extra electricity, and substation 7, 8a, 9a, 12 are more likely to have export potential. However, since most substations have negative average values, there are huge gaps between production and loads. Thus, external grid is necessary. In winter, average numbers of all substations are negative and the gap is larger than that in summer. But substation 3 and 9a are with positive range, which represents that these two substations possibly export electricity even in winter in a certain condition.

**Table 4:** Average and range of difference between production and loads in two seasons of all substations (unit: kW).

station	Summer		Winter	
	Average	Range	Average	Range
1a	−38.56	[-236.96, 47.10]	−177.96	[-390.33, −166.02]
1b	−45.90	[-160.51, −0.07]	−120.56	[-264.40, −112.97]
2a	−7.55	[-494.58, 189.61]	−337.17	[-836.94, −265.57]
3	−81.86	[-139.75, −41.12]	−104.86	[-234.64, 17.84]
4	−76.22	[-512.09, 268.65]	−317.88	[-810.78, −196.39]
5	−134.85	[-1268.38, 7.01]	−392.25	[-1563.22, −168.56]
6	−98.79	[-558.05, 121.58]	−508.47	[-973.09, −444.52]
7	52.27	[-567.82, 338.16]	−452.95	[-883.72, −261.14]
8a	15.97	[-396.55, 309.69]	−257.90	[-603.64, −169.30]
8b	−248.32	[-589.52, 17.00]	−359.28	[-840.81, −324.83]
9a	160.27	[-25.17, 273.59]	−20.11	[-81.57, 53.66]
9b	−107.21	[-459.52, 235.82]	−814.01	[-1466.38, −657.94]
10	−258.90	[-717.84, −65.35]	−167.86	[-1160.51, −26.67]
11	−162.85	[-876.80, 125.53]	−76.11	[-1393.20, 0.18]
12	32.74	[-530.72, 259.26]	−454.12	[-898.88, −284.01]
13	−560.13	[-1109.09, −405.91]	−573.69	[-1282.42, −452.08]
14	−162.73	[-790.87, 69.94]	−575.43	[-1256.86, −506.78]
15a	−137.97	[-579.15, 48.54]	−332.56	[-807.27, −307.43]
15b	−171.85	[-805.58, 99.17]	−462.66	[-1122.68, −427.70]

Full use of all the available rooftop area in Hammarby causes a line overloading problem in some of the substations. Based on Fig. 9, the problem arises in 11 substations out of 19 in total during the year, but the frequency varies a lot. Among these substations, the problem mostly happens between 200 and 700 times annually. The situation is more severe in substation 7, 8a and 13. Among these three substations, substation 13 has the highest frequency 2358 times in one year followed by substation 7. There are two substations with the problem less than 100 times-substation 6 and 15b, and only 6 times for substation 15b.

**Fig. 9:** Annual line overloading situations of each substation.

In the influencing area of each substation, not all the buildings will have line-overloading problem, nor does it happen every month. Fig. 10 presents more details of line-overloading problem specifically at building and month. The colors of the cells represent the frequency difference, with green as low and red as high. It is observable that, in general, line-overloading problems in those substations with higher frequency arise in more months. In addition, in the influencing area of both substation 7 and 13, there is one building where line overloading occurs all the months. The peak value in summer is more than 200 times in one month. That is why substations 7 and 13 have the highest frequency over the year. This might result from the huge rooftop area for single building. The grid-integration lines are the same for all the buildings, there is a thresholds value for the line and corresponding maximum power output value. Thus, buildings with large rooftops are more likely to reach or transgress the thresholds of the lines even with smaller irradiation. The available area of building 7- [1] and 13- [1] are much larger than the thresholds. Unlike substation 8a and 13, substation 4 also has 3 buildings occurring line overloading but the total value remains small. This is because the buildings of substation 4 are uniform and the area is much closer to the thresholds value.

**Fig. 10:** Line overloading situations of the buildings in each month (Unit: hour).

There is more line-overloading situation reported from May to July. And all buildings with line overloading situation report the problem in May and June. Available solar irradiation in Sweden locating at high latitude is much higher in summer. Therefore, even though the rooftop area is not such big; it is also possible to reach the thresholds. In this study, the weather data comes from the year 2020 so there might be contingency. For example, the weather in December is mostly cloudy with low available irradiation, which leads to the much lower frequency in December compared to January. However, the overall trends are similar.

As loads data are aggregated by substations, the line loading keeps at low level without PV systems. When integrating with PV systems, the line loading rises dramatically. Table 5 presents the maximum monthly average value of the line loading of each substation in scenario 1. If the value is larger than 100%, it is regarded as line overloading. These numbers correspond to the occurrence of line overloading situation in Fig. 10. They are mostly between 100 and 200%, but the maximum one is almost 348% which is more than twice higher than the thresholds. Due to delf-consumption, the transformer loading of each substation generally decreases. Table 6 shows this reduction in transformer loading in scenario 1.

**Table 5:** Maximum line loading each month at each substation in scenario 1 (unit: %).

	Jan	Feb	Mar	Apr	May	Jun	Jul	Aug	Sep	Oct	Nov	Dec
**1a**	46.45	53.50	62.53	62.37	67.78	67.66	62.59	60.89	57.99	50.20	44.06	36.11
**1b**	11.72	13.27	15.20	14.95	15.99	15.97	14.55	14.19	13.64	11.96	11.08	9.16
**2a**	51.82	58.14	70.48	76.78	82.85	84.10	81.09	78.28	71.52	58.69	47.85	38.60
**3**	22.45	27.98	31.50	33.22	33.67	34.99	34.45	32.31	31.37	26.77	23.87	15.89
**4**	66.89	89.04	110.11	118.52	132.22	131.26	128.78	120.78	114.11	89.57	68.17	49.82
**5**	65.16	83.65	101.81	110.64	120.10	121.23	117.93	112.64	104.98	84.19	65.52	53.27
**6**	51.48	72.82	91.33	99.73	108.33	109.96	107.18	102.50	92.93	73.56	52.19	38.11
**7**	153.25	203.69	244.74	265.06	286.35	289.12	279.88	269.51	248.61	205.27	154.73	112.59
**8a**	92.79	124.92	151.52	164.55	179.38	180.08	174.76	168.05	155.16	126.07	95.06	68.78
**8b**	61.79	71.24	80.98	83.70	86.00	88.69	81.49	82.30	79.08	69.06	55.26	41.77
**9a**	95.73	128.27	155.18	168.16	182.37	183.90	177.72	171.32	157.60	129.13	97.14	70.61
**9b**	69.89	92.79	111.78	121.00	130.85	132.03	127.54	123.09	113.33	93.35	70.43	51.36
**10**	52.27	65.42	76.99	82.42	87.72	89.64	85.11	88.13	79.11	67.16	50.72	40.02
**11**	53.38	68.79	81.49	87.13	94.87	99.13	96.27	93.98	84.63	69.18	56.97	40.04
**12**	63.65	74.05	86.81	89.12	98.03	94.27	89.92	87.72	83.50	71.22	59.88	47.87
**13**	178.52	233.70	294.11	309.79	345.65	347.91	334.51	317.03	294.99	231.32	180.60	126.80
**14**	73.45	84.36	96.66	98.56	104.17	104.33	100.75	96.94	91.89	79.65	65.45	54.90
15a	64.74	86.73	104.75	113.62	122.90	124.17	119.94	115.62	106.39	87.31	65.37	47.36
15b	67.24	77.56	89.52	94.69	102.15	101.53	98.10	95.86	88.88	76.41	65.13	50.18

**Table 6:** Maximum monthly difference of transformer loading at each substation in scenario 1 (unit: %).

	Jan	Feb	Mar	Apr	May	Jun	Jul	Aug	Sep	Oct	Nov	Dec
**1a**	13.98	18.69	22.57	23.16	24.72	24.80	20.40	21.45	21.40	18.68	14.11	10.16
**1b**	17.44	23.61	28.62	31.15	33.77	33.66	31.61	31.44	29.13	23.81	17.63	12.58
**2a**	28.29	36.90	43.86	44.30	37.47	37.57	32.96	37.77	39.07	34.58	28.52	20.60
**3**	3.75	5.03	6.12	6.65	6.79	7.29	7.03	6.78	6.23	5.09	3.76	2.73
**4**	38.17	49.96	56.78	54.69	57.96	63.66	51.92	55.60	55.55	50.31	34.17	21.84
**5**	20.30	27.06	32.48	34.96	37.31	37.56	35.58	35.49	32.58	27.22	20.47	14.78
**6**	26.69	35.35	42.06	44.66	44.92	45.79	40.37	41.32	40.87	35.51	26.89	19.43
**7**	40.25	51.04	55.10	52.55	51.06	51.12	44.36	49.56	50.09	45.05	40.39	29.64
**8a**	46.23	60.90	68.64	69.66	68.39	63.59	56.76	65.05	63.43	59.55	43.61	33.83
**8b**	35.57	47.40	57.08	61.54	64.00	66.62	61.34	61.30	57.12	47.58	35.65	25.90
**9a**	9.69	21.16	31.30	33.32	37.23	38.59	36.76	34.64	31.41	19.71	12.94	8.32
**9b**	28.73	40.81	50.86	55.74	60.96	61.59	59.21	56.85	51.68	41.11	29.02	18.99
**10**	15.70	20.91	24.97	27.17	28.81	29.54	28.09	27.89	25.34	21.06	15.84	11.47
**11**	37.00	47.19	55.41	60.43	52.08	68.58	64.34	65.37	56.34	42.35	37.41	26.91
**12**	38.53	51.50	61.50	64.02	61.54	45.96	53.73	57.79	52.11	51.13	38.86	28.04
**13**	18.84	24.80	29.44	31.40	33.15	34.25	31.93	31.69	29.68	24.92	18.49	13.77
**14**	41.43	55.46	66.91	72.15	75.07	76.51	72.20	71.33	67.48	55.66	41.73	30.11
**15a**	35.65	47.52	57.16	60.49	64.38	63.12	55.27	60.15	57.07	47.79	35.94	26.02
**15b**	45.65	60.99	73.74	79.62	86.12	84.79	80.97	80.81	74.52	61.35	46.00	33.20

#### 3.1.2 Scenario 2

In order to avoid line-overloading problem, the PV system is re-sized in scenario 2. Those buildings with the problem should reduce the area for PV installation. Table 7 presents the maximum line loading value of each substation in scenario 2. The table validates that the line overloading problem is avoided. Compared with scenario 1, transformer loading increases in some substations since the PV installation is modified. Table 8 shows this difference.

**Table 7:** Maximum line loading each month at each substation in scenario 2 (unit: %).

	Jan	Feb	Mar	Apr	May	Jun	Jul	Aug	Sep	Oct	Nov	Dec
**1a**	46.45	53.50	62.53	62.37	67.78	67.66	62.59	60.89	57.99	50.20	44.06	36.11
**1b**	11.72	13.27	15.20	14.95	15.99	15.97	14.55	14.19	13.64	11.96	11.08	9.16
**2a**	51.82	58.14	70.48	76.78	82.85	84.10	81.09	78.28	71.52	58.69	47.85	38.60
**3**	22.45	27.98	31.50	33.22	33.67	34.99	34.45	32.31	31.37	26.77	23.87	15.89
**4**	54.59	69.22	82.14	89.02	98.70	97.84	96.13	90.57	85.17	69.69	51.40	37.32
**5**	55.12	66.95	81.67	88.84	96.51	97.43	94.93	90.46	84.56	67.39	55.40	45.82
**6**	46.16	64.28	80.47	87.87	95.47	96.90	94.46	90.32	81.88	64.92	46.65	36.71
**7**	69.75	78.47	89.44	92.07	97.84	99.07	92.69	93.87	86.84	73.36	62.25	50.66
**8a**	51.61	69.58	84.46	91.76	99.13	99.45	97.54	93.76	86.59	70.24	52.97	38.29
**8b**	61.79	71.24	80.98	83.70	86.00	88.69	81.49	82.30	79.08	69.06	55.26	41.77
**9a**	46.94	63.35	76.86	83.32	90.55	91.25	88.24	85.00	78.18	63.81	47.93	34.77
**9b**	52.36	69.77	84.27	91.33	98.89	99.80	96.35	92.93	85.45	70.20	52.78	38.34
**10**	52.27	65.42	76.99	82.42	87.72	89.64	85.11	88.13	79.11	67.16	50.72	40.02
**11**	53.38	68.79	81.49	87.13	94.87	99.13	96.27	93.98	84.63	69.18	56.97	40.04
**12**	63.65	74.05	86.81	89.12	98.03	94.27	89.92	87.72	83.50	71.22	59.88	47.87
**13**	66.10	67.56	68.86	70.54	75.23	77.92	71.24	70.84	70.20	67.14	66.46	66.10
**14**	65.87	75.01	85.83	87.28	91.80	91.97	88.75	85.47	81.11	70.55	58.32	49.35
**15a**	60.85	70.50	82.94	90.04	97.45	98.49	95.12	91.65	84.28	69.67	59.07	45.40
**15b**	65.94	75.90	87.42	92.42	99.69	99.05	95.71	93.55	86.75	74.65	63.82	49.25

**Table 8:** Difference of transformer loading between sccenario 1 and 2 (unit: %).

	Jan	Feb	Mar	Apr	May	Jun	Jul	Aug	Sep	Oct	Nov	Dec
**4**	4.51	5.61	6.04	1.81	3.30	4.80	1.16	3.07	4.33	5.66	2.47	0.29
**5**	1.78	2.32	2.68	2.77	2.68	2.65	2.77	2.77	2.69	2.33	1.80	1.32
**6**	0.68	0.87	1.01	1.05	0.40	0.57	0.13	0.77	0.70	0.86	0.69	0.50
**7**	11.09	12.33	8.60	6.04	2.24	1.15	0.47	3.91	5.20	6.69	10.99	8.36
**8a**	7.65	9.58	7.41	6.03	3.64	2.62	1.22	3.88	2.83	8.07	4.92	5.54
**9a**	0.13	6.39	7.93	8.28	9.36	9.33	9.00	8.51	8.12	6.53	5.06	0.83
**9b**	2.02	2.66	3.18	3.43	3.69	3.72	3.60	3.48	3.22	2.68	2.04	1.50
**13**	11.47	14.82	17.31	18.26	19.01	19.82	18.12	18.32	17.44	14.88	11.00	8.42
**14**	1.73	2.28	2.70	2.78	1.16	2.23	2.69	2.33	2.61	2.28	1.74	1.28
**15a**	1.34	1.73	1.98	1.47	0.98	1.83	0.58	0.73	1.62	1.73	1.35	1.00
**15b**	0.04	0.02	0.00	0.02	0.03	0.03	0.01	0.02	0.01	0.02	0.03	0.04

Fig. 11 presents the summary of area reduction in each substation. Those with a higher frequency of line overloading present larger area reduction. But the reduction is little relative to the original area. PV production is still positively relative to the area, and it will also accordingly. The total area reduces by roughly 9000 square meters and correspondingly the total production decreases to about 9000 MWh.

**Fig. 11:** Areas and production in scenario 2.

Fig. 12 demonstrates the relationship among solar fraction, self-consumption and self-sufficiency in scenario 2: Fig. 12a shows the relationship between solar fraction and self-consumption and Fig. 12b shows the relationship between solar fraction and self-sufficiency. The solar fraction is at a low level for most of the substations, less than 20%, except substation 9a with more than 90%. For the stations that area keeps the same, the value remains same, such as station 3. However, for modifying the rooftop area, the value is smaller compared with scenario 1. For example, for substation 13, solar fraction drops from 7% to 3%, as well as substation 9a from 117% to 91%. This is because production decreases due to smaller areas for PV installation.

**Fig. 12:** Difference between scenario 1 and 2: (a) self-consumption and solar fraction; (b) self-sufficiency and solar fraction.

Similarly with scenario 1, self-consumption value keeps at high level for the majority of substations. Since the total production is smaller while the loads are same, self-consumption for scenario 2 is slightly larger than that of scenario 1. However, as solar fraction changes a lot, the distribution of dots is quite different with scenario 1. The exception is substation 9a where the self-consumption is less than 40%. Most of the PV production is not used for loads but “wasted” within the current situation. This part of extra electricity is potential to export.

Self-sufficiency is positively related to solar fraction. The distribution of the dots is similar to that of scenario 1, but the value is a little smaller. Unlike solar fraction, the influence on self-sufficiency is not significant with increasing solar fraction, approximately 1%–3%. Even if PV generation decreases, the loads can be satisfied as scenario 1. For instance, when the decrease is relatively small during the periods that production is higher than the loads, PV production in scenario 2 maintain higher than the loads and the self-sufficiency would not change. Another reason is that the difference in the total amount of electricity is relatively small compared with total loads. Therefore, this ratio is not significantly changed.

The export potential presented in Fig. 13 presents the export potential of all substations and the relationship with self-consumption. In scenario 2, there are also 18 substations with export potential except substation 13. Substation 9a is still the main contributor to electricity export, but this part of electricity reduces to less than 180 MW h. The export potential of the rest substations is lower than 80 MW h. Basically, the relationship of self-consumption and export potential is similar. But the export potential is smaller and self-consumption is higher for some dots, which leads to a difference at the distribution within the figure. This is due to rooftop area reduction. The changes on self-consumption in substation 7 is most evident, increasing from 89% to 97%, while the greatest variation occurs in substation 9a followed by substation 7.

**Fig. 13:** Exported energy and self-consumption of each substation for scenario 2.

Fig. 14 summarizes the comparison of scenario 1 and 2 from different perspectives. The area for PV installation in scenario 2 is about 90% of that in scenario 1, as well as the total PV production. Besides, as the total production is lower, the modification influences the amount of electricity used for self-consumption and increases the dependence on external grid. The largest impact is on the potential of energy export compared with former two (about 92% of the maximum potential). The potential decreases to around 70% of maximum one. When the total PV modules diminish, the period when the production is greater than loads becomes even less and the gap between production and loads becomes narrow. Therefore, the energy export potential tails off significantly. On the other hand, a larger proportion of electricity produced is used to satisfy the load demands (94.1% vs. 85.2%) so the impact is much smaller.

**Fig. 14:** Comparison of feasible and maximum potential of the system from multi-aspects.

### 3.2 Economics

The costs of both scenarios are listed in Fig. 15. Fig. 15a shows the condition without subsidy, while Fig. 15b represents the situation with subsidy provided by the government. The majority comes from CAPEX and OPEX is relatively small. Since the system for scenario 1 requires more components, CAPEX and OPEX is higher than scenario 2. It is noted that political support of capital reduction has a strong influence on the total initial costs, making the option more attractive to investors.

**Fig. 15:** Impact of subsidies on cost for both scenarios: (a) Without subsidy; (b) With subsidy.

Since the system price varies among different sizes, size estimation can influence the total CAPEX. The size of PV system is measured by each building separately in this study as shown in Fig. 15. However, the buildings are aggregated with substations within in the influencing areas. Another option is to size by substations. Fig. 16 presents the comparison of CAPEX with system size categorized by buildings and substations. Scenario 1.1 and 2.1 refers to calculation categorized by buildings, same as conditions in Fig. 15; whereas scenario 1.2 and 2.2 refers to calculation categorized by substations. According to Fig. 16, calculation by substations can significantly reduce the CAPEX compared with calculation by buildings, due to lower system price of larger size of systems. When aggregated with substations, the cost difference between scenario 1 and 2 becomes larger. It represents that scenario 2 benefits more from this change. Lower CAPEX corresponds to a higher possibility of profitability, and it is more attractive for consumers.

**Fig. 16:** Comparison of different system price calculation.

Integration with PV systems reduces costs on electricity fees and earns from selling extra. Thus, variation of electricity price would influence the total benefits of the system. Fig. 17 calculates indicators of benefits for both scenarios with different electricity prices. Fig. 17a shows the comparison of indicators in scenario 1 and Fig. 17b presents the results of scenario 2. Electricity price of 2020 is relatively low, while that of 2021 is at a high level. Since the majority of electricity generated is for self-utilization within the influencing area, the saving due to consumption reduction is dominant of total saving (approximately 95%). The gains much depends on the electricity price. TB of 2021 is approximately twice as much as that of 2020. Scenario 1 earns more than scenario 2 in both conditions due to higher generation.

**Fig. 17:** Potential benefits for both scenarios with different electricity price: (a) scenario 1; (b) scenario 2.

Table 9 summarizes NPV prediction in different conditions, including variation on electricity price (2020 or 2021), subsidy (with-Y or without-N) and size measurement (by building-B or substation-S). The NPV values overall do not remain positive for all situations. Electricity price has a large impact on NPV values and profitability of the system. With low electricity price, the system consistently results in negative NPV values. However, with high electricity prices, the system is much more likely to get positive ones. Financial support from the government and size measurement also plays important roles. When a system is sized by buildings, NPV can only be positive with the CAPEX subsidy. Similarly, without subsidies, positive NPV is obtained with size measured by substations.

**Table 9:** Summary of NPV with different conditions.

	Electricity price	subsidy	Size measurement	NPV
**Scenario 1**	2020	Y	B	−48.40
			S	−17.64
		N	B	−65.90
			S	−30.99
	2021	Y	B	11.19
			S	39.86
		N	B	−6.31
			S	26.51
**Scenario 2**	2020	Y	B	−49.47
			S	−16.37
		N	B	−66.38
			S	−28.58
	2021	Y	B	4.52
			S	35.73
		N	B	−12.38
			S	23.53

In general, scenario 1 performs better than scenario 2 according to Table 9, due to greater production in scenario 1. But there are exceptions: when electricity price is low, and system is sized by substations, the NPV value of scenario 2 is larger than that of scenario 1. Because the PV panels are reduced, system in scenario 2 is in smaller size, which leads to higher system price. When aggregated with substations, savings for scenario 2 are higher. Besides, the difference in TB is small with low electricity price. As CAPEX domains the total costs, CAPEX saving is larger than the difference in TB. Thus, scenario 2 has better performance in this certain condition.

In short, this study evaluates the potential of urban distributed PV systems. 4 technical indicators and 2 economic indicators are mainly measured and analyzed. Based on the results above, the indicators are related to each other, and they will have different impacts on the size of the PV system as well as solar generation potential. However, it is unlikely to achieve that all the indicators are optimized at the same time, there might be some trade-off required for the final decision. With different goals, the PV size might vary. In order to achieve 100% renewables by 2040, the PV production should be maximized then total benefits might be sacrificed. However, customers and investors care more about prices and profits, so total benefits and NPV should be priority.

The approach in this study is quite general. With different requirements, there would be various combinations of different aspects. This paper involves the combination of space, grid, irradiation and economics. The changes in these characters can lead to different conclusions. The equations may slightly change but the methods in general are similar. The approach could be used for other regions with different conditions as long as local data is accessible.

## 4 Conclusions

The paper evaluates and analyzes the potential of rooftop PV systems considering spatial limitation, infrastructure conditions and economics in a Swedish context. A real test case referring to a district named Hammarby is developed and simulated. Both technical and economic aspects are estimated through several indicators to provide a comprehensive overview of urban solar potential.

According to the results, the rooftop PV systems do have considerable power potential in Sweden: annually more than 10 000 MW h with maximum PV installation and more than 9000 MW h with infrastructure limitations. The system contributes to renewable transition by reducing dependence on external grid that may come from fossil fuels. Since there are no more land requirements for the installation, it is also one solution for satisfying future increasing electricity demands and relieving the pressure of grids. However, the integration of the PV system cannot totally fulfill the demands in the district. There is a huge gap between production and loads. Also, the current infrastructure constrains fully utilizing the rooftop which also restricts the transitions. Besides, the PV generation relies on weather conditions and the output is unstable day and night or in different seasons. Thus, external grid is still necessary.

From the economic aspects, the CAPEX of the systems domains the total costs. The systems with maximum PV installation generally have better economic performance. The economic feasibility of the system is heavily sensitive to the electricity prices, size measurements and financial support from the government. And electricity price has the largest impact on the economic feasibility. PV system aggregated by substations can also significantly reduce the costs and provides huge possibility of economic feasibility.

In the future, with better materials for the panels with higher efficiency and mature techniques of manufacturing and installation, the costs can be further lower. With growing population along with increment of energy demands, it is urgent to make rational use of all available resources. This research validates the feasibility of this kind of system applied in high latitude areas and can be a reference to extend to other districts with similar conditions.

## Author contribution statement

Tianqi Ruan: conceived and designed the experiments; performed the experiments; analyzed and interpreted the data; contributed reagents, materials, analysis tools or data; wrote the paper. Monika Topel: conceived and designed the experiments; analyzed and interpreted the data; contributed reagents, materials, analysis tools or data; Wujun Wang, Bjorn Laumert: conceived and designed the experiments; contributed reagents, materials, analysis tools or data.

## Data availability statement

Data included in article/supplementary material/referenced in article.

## Declaration of competing interest

The authors declare that they have no known competing financial interests or personal relationships that could have appeared to influence the work reported in this paper.
